# Neighboring Algorithm for Visual Semantic Analysis toward GAN-Generated Pictures

**DOI:** 10.1155/2022/2188152

**Published:** 2022-09-23

**Authors:** Lu-Ming Zhang, Yichuan Sheng

**Affiliations:** ^1^Key Laboratory of Crop Harvesting Equipment Technology of Zhejiang Province, Jinhua Polytechnic, Zhejiang, Jinhua 321007, China; ^2^Hithink RoyalFlush Information Network Co., Ltd., Zhejiang, Hangzhou, China

## Abstract

Generative adversarial network (GAN)-guided visual quality evaluation means scoring GAN-propagated portraits to quantify the degree of visual distortions. In general, there are very few image- and character-evaluation algorithms generated by GAN, and the algorithm's athletic ability is not capable. In this article, we proposed a novel image ranking algorithm based on the nearest neighbor algorithm. It can obtain automatic and extrinsic evaluation of GAN procreate images using an efficient evaluation technique. First, with the support of the artificial neural network, the boundaries of the variety images are extracted to form a homogeneous portrait candidate pool, based on which the comparison of product copies is restricted. Subsequently, with the support of the *K*-nearest neighbors algorithm, from the unified similarity candidate pool, we extract the most similar concept of K-Emperor to the generated portrait and calculate the portrait quality score accordingly. Finally, the property of generative similarity that produced by the GAN models are trained on a variety of classical datasets. Comprehensive experimental results have shown that our algorithm substantially improves the efficiency and accuracy of the natural evaluation of pictures generated by GAN. The calculated metric is only 1/9–1/28 compared to the other methods. Meanwhile, the objective evaluation of the GAN and human consistency has increased by more than 80% in line with human visual perception.

## 1. Introduction

Generative adversarial networks (GANs) [1] are deep visual processing models. In 2014, they gained a high reputation in the fields of visual processor and feature language programs. In addition to producing extraordinary realistic images [2], GANs can also be utilized in semi-supervised learning [3], concept in painting [4], image-to-image translation [5], and other fields of simulation tasks. GAN Variety Image Quality Assessment [6] is the reason for evaluating actors through GANs and attempting to get the image warp in the process of image generation [7, 8]. Whether it affects the observer's cue acquisition and objective perception is unknown. Although variable GAN models have been designed, the visual appearance produced by different GAN modalities is strange. That is, not all fertility images experience the demands of specificity requirements. The most pervasively used GAN evaluation metrics, such as Inception Score [9], Fréchet Inception Distance [10], and Mode Score [11], all focus on the evaluation of generative models. However, they cannot perform an uncompounded generative operation. Subjective character evaluations of pictures generated by GAN models are not only a waste of human fate and significant expediency, but also flame inefficient. We in this fictitious address a peculiarity-assessment sequence for generating GAN picture wherein the pipeline is robot-like, outward, and competent. We take the properties of images produced by GAN modalities. In the aspect of personate, quality assessment techniques for breed similarity are proposed from two different perspectives: (1) knowledge-based growth image quality assessment methods and data-based conformation attribute assessment methods [6]. A feature evaluation method for generative images based on the learning-necessary convolutional neural network structure [12] is deployed. The network bifurcation returns the quality scores of the growing images. We further use a variety of binary classifiers as regressors to generate actor quality through half-check scholarship research evaluation, models, and databases. (2) The data-guided learning algorithms for evaluating the attributes of reproduced actors can be decomposed into parameter methods and parameter-free ones. The former applies a Gaussian mixture model to capture the likelihood distribution of the real data and subsequently generate images by estimating the probability distribution toward the real data. However, the density of model selection cannot well capture complex data distributions. In contrast, distribution-free methods obtain the probability of generating pictures by predicting the variance between the generated idol and its *K*-nearest boundaries. This is a process guided by large space occupancy and computational cost. And it is expensive and inefficient for algorithmic program management.

Most of the existing picture quality evaluation algorithms are designed for grayscale images, such as Structure SIMilarity [3] and gradient magnitude similarity deviation [4]. Comparatively, the agreement of the picture conception is relatively less satisfactory in property evaluation. It means to appraise the flush similarity violent supported on the scattered manifest and reconstruction residuals [5]. Then, we use an overcomplete similarity dictionary to guide conventional excuse portraits to display reference similarity and warped similarity. And it invents two feature plane spheres to measure the portrait architecture and color metamorphosis. Meanwhile, it computes the reconstruction residuals to assess contrast bias in replicas, and further generates photometric similarity to successfully document the final quality of camouflaged portraits. Reference [6] proposed an algorithm to optimize the similarity mapping with appearance similarity variance as an unbiased function. The algorithm program solves the problem of different optical artifacts in the images generated by the traditional color scale corresponding algorithm program. Also it provides a modified color image competition index that validates the predictive role of color image quality. It was also proposed to converse a multi-scale method that converges on false-concept quantitative phantoms (competition between advertising images and their copies) and further addresses blush notification and pigment teaching sedimentation by spectral statistics of grayscale images. This model is built upon the selectivity of human vision system (HVS) and hierarchical propositions. It is intended to support an image professional evaluation algorithm on superpixels [8] that calculates the supported photometric luminance, chrominance, and gradient similarities on perceptually meaningful superpixel image patches. Finally, the interleaving complexity is leveraged as the moment function of the pooling layer to calculate the consistency based on the target score.

Regarding the performance of the trained model, we in this article proposed a competitive rating scheme for variety of images based on the nearest neighbor (NN) algorithms. This method aligns the proximate neighbor algorithm rules with the *K* to NN algorithm program. It can further shorten the measurement speed of appearance similarity while ensuring the accuracy of quality estimation. The neural bifurcation extracts the feature notification of the generated image and the real image. The second is to utilize the artificial neural network (ANN) algorithm to receive a real display, that is, consistent with the growth map to produce a similar image. Finally, the *K*-nearest neighbors (KNN) algorithm is utilized to eliminate the recurrence in the similarity candidate decoy. The calculation is based on the most similar pictures. Experimental results have shown that the method proposed by us can effectively avoid the contradiction between the calculation speed and the fidelity of the generated image by leveraging the quality evaluation mode.

## 2. Related Work

Generally speaking, our proposed method is closely related to three topics in machine learning and computer vision.

### 2.1. Visual Quality Prediction

Through the decomposition of image features, it is studied to determine whether the distortion of image attributes in the process of visual information acquisition, transmission, compression, etc. Distorted images will affect observer's enlightenment acquisition and objective loss. From the method point of view, it can be divided into subjective and objective image quality evaluation techniques. For appearance-based quality evaluation methods, the objective image quality evaluation methods can well support human visual perception and understanding of each image. This is obtained to score the quality of each picture. The commonly used visual quality prediction methods maintain the normal objective record and the average objective account variance. The mathematical calculation model supports the unbiased prediction of the quality evaluation method.

Determined by whether there is a corresponding related image, the prediction can be divided into three categories: full-view image property evaluation, semi-relational image level evaluation [12–14], and ignoring portrait temper evaluation [15]. The quality evaluation of the entire allusions copy is effective in evaluating these attributes. Here, the active images are used as references. Pervasively used methods include input squared error, vertex signal-to-noise ratio [16], and structural parity [17]. Semi-reference image quality assessment is to leverage partial information from aspect replicas to assess whether an image is standard or not. Popular methods include methods supported by fresh show shapes [18, 19], simple wavelet real estate statistics examples, and multidistribution geometric analysis support method. Both methods evaluate visual perceptual attributes by maintaining part of the characteristic information of the picture. The difference is that the quality evaluation of the unnatural images focuses on images generated by the GAN model rather than natural pictures. Meanwhile, pictures propagated by the GAN may contain some particular distortions for the generative model. Quality assessment of unreferenced images is completely different from the quality evaluation in an ideal reference picture and is the most pervasively used quality assessment tool. In practice, an analog analysis model should be established on the basis of image statistical characteristics. In this way, the appearance-based image quality evaluation results are calculated by leveraging the visual characteristics of the image to be evaluated.

### 2.2. NN Algorithm

NN algorithm procedures are widely applied in the fields of textbook information recovery, image information suspicion, and so on. The starting point of NN's work is addicting a scaling operator that contains dataset and target data. It then discovers the relationship between the dataset and target data. The most typical data for this type of operation: KNN is a supervised learning algorithm speak by Cover and Hart in 1967. The keynote technique of KNN is to find the instructive set and hypothesis based on a stated alienation limit, and further foreshow the *K* university samples that are closest to the pattern on the *K* “adjacent” advice.

Common reckoning methods include Euclidean distance, Manhattan opposition, and Minkowski reserve. Closed farthest neighbor (ANN) algorithm can solve this problem. NN and KNN suffer from the problem of calculating behavior validity and unexpected range. ANNs are assembled with the intent to obtain local data that might be the neighbors of the data to be normalized, rather than keeping only the most probable neighbors of the entire data to be distinguished. We can improve the computation scheduling and preserve loading space while breaking accuracy within acceptable limitation. The ANN generally adopts the crushing method, the wood method, the vector quantization method, and the NN graph processing. It can further improve the distance calculation ability by shortening the distance calculation time. Locality sensitive hashing (LSH) is a typical algorithmic procedure in ANN. The basic concept of LSH is similar to the idea of space domination transformation. If pairwise data points are similar in the real data distribution, their checksums are also the same. If the two data are unsimilar, there is still no difference after the hashing step.

### 2.3. Color Descriptors

Computer network(CN) [12] can be treated as a good appearance descriptor given a GAN-produced image. This technique uses an 11-dimensional probability vector to describe similarity. Each integral of this vector represents that blush belongs to 11 colors, which can be accurate and intuitive. Moreover, it can be described semantically and probabilistically. What makes the CN effective is the practicality of the semantic description of the feature, which takes a black-box way of characterizing the ingenuity of human color perception. This wallpaper uses CN to build an example of color appearance grades that will correlate to the appearance and each pixel inside the generated image. We map the CN credibility vector and further calculate the discrepancy between two vector distributions by leveraging the Wasserstein reserve to enhance the perceptual color difference between pairwise similarities. We subsequently convert attractive portraits and distorted images to each channel [13]. The self-reliant adversarial hidden hawser (Opponent Color Space) intensifies to represent its glittering channels. And mount form that can represent stageplayer form information are quotation. Since HVS is more tender to luster vary than to excuse, and hominal apprehension of appearance is secretly related to radiance, we increase the brightness of bifurcations. Multiple features are then leveraged as the complements. Visual saliency is treated as the natural fraction used as the load cosecant to dominate in pooling stagecoaches. Experimental validation on several hotel datasets demonstrated that conversation examples can outperform multiple valuation issues.

## 3. Our Proposed Method

Based on the concept of image quality evaluation, we in this work calculates the image features motivated by predicting the feature similarity between the fertility image and the real image. Afterward, we evaluate the fertility image accordingly. The process can be elaborated as follows. The image features are converted into binary vectors through the LSH algorithm in order to shorten the angle and spatial entanglement. Subsequently, the neighbors of the generated image are successfully supported on the ANN algorithm so as to form a consistent similarity confirmation pool. This can reduce the amount of computation. Finally, based on the support of KNN algorithm rules, similar appearance candidates with the most similar features to the generated image are calculated in the pond. Meanwhile, the GAN-generated image attributes are calculated to reduce the computational burden.

As shown in the dotted box in the following, for the real similarity data plant *D*, the similarity form is essentially the feature vector data adapter *M* of the real image calculated through convolution neurons. This is based on the form extraction function *F*(·), then the shape vector *m*_*i*_ = *F*(*i*) of the *i*th image in the actual image dataset. Note that, herein, *i* = 1, 2, ⋯, *N*,*M* = {*m*_1_, *m*_2_, ⋯, *m*_*N*_}. For the *j*th feature vector *m*_*i*_ of the *i*th image form *m*_*ij*_, we use the gate binarization activation cosecant *H*′ to calculate the two summaries *h*_*ij*_ corresponding to *m*_*ij*_, if *m*_*ij*_ > 0, then *h*_*ij*_ = 1, else *h*_*ij*_ = 0 where *j* = 1, 2, ⋯, *s*, and *s* denotes the many forms of the image shape vector *m*, *h*_*i*_ = {*h*_*i*1_, *h*_*i*2_, ⋯, *h*_is_}.

The reciprocal of the binary star-encoded data hinders the Kerçek image shape vector dataset *M* can be expressed as *H* = {*h*_1_, *h*_2_, ⋯, *h*_*N*_}. The extracted visual features of the real image dataset and their corresponding binary codes are preserved in the form of H5 (Hierarchical Data Format, HDF5) files. Moreover, the data is stored in a hierarchical structure unique to the file system to calculate different representations of data storage and faithful bursting. Here, we present the flowchart for calculating the binary encoding of conceptual features.

Here, the Wasserstein Opposition is leveraged to evaluate the contention between the CN similarity vector focusing on similarity and warped similarity. It is also used to measure the perceived color difference between the two images. First, the appeal image and the corresponding power-grabbing portrait are re-worn mapping tables only according to [12]. Each pixel in is mapped to an 11-dimensional CN similarity vector, and then we are interested in the distance between the two vectors to broaden our understanding of similarity differences. How to measure the divergence between two confidence vectors (distributions) is a difficulty. Common methods are the Kullback–Leibler (KL) divergence and the Wasserstein constraint, where the Wasserstein ritual, also known as Earth Movement Distance , is the minimum attention that must be paid to convert one histogram into another. Wasserstein constraints are mathematically improved over KL divergence. They can still account for the coldness of two distributions even if their back resistances do not interlap or ride very contracted. In this road, Wasserstein dissimilation is a degree of the diversity between two CN likelihood vectors: CND_*i*_ = WSY *f*_r_ ( *i* ) + *Y* *f*_d_ ( *i* ), where *f*_r_ denotes the attention image and *f*_d_ means the distorted portrait. *i* represents the “image roof” index, *Y*(·) represents the mapping of appearance pixel values to CN chance vectors, WS(·) represents the Wasserstein distance operator, and CND denotes the species name dissimilation.

For certain distortions that may be contained in GAN-generated images, such as exemplary and unreasonable structures, convolutional neural networks are leveraged for shape extraction. This results in image features Mikoyan that can adequately represent the generated image *I*_g_. The dual code *hI*_g_ is similar to Mikoyan, which estimates the Hamming coldness digest *h*_*i*_ ∈ *H* between chaise and ground truth basis 2, which is dominated by a similar pool of image licenses *P*. If the Hamming constraint between fiddle and hi is frowned more than Limen *T*, then *h*_*i*_ corresponds to the actual similarity added to the similarity idol trial pool *P*, *P* = {*i*_1_, *i*_2_, ⋯, *i*_*c*_} and *c* denotes the true appearance of the experience requirement enumeration. Get the fitted form vector of the pictures in the similar image capability pool *P* from the shape vector dataset *M*. The quality of this disembodied propagating image is a duration measured by the similarity between the generated image and the nearby true similarity in high-dimensional form. Moreover, the similarity between the grown actor and the royal appearance is calculated by cosine similarity. Assuming the feature vector Mikoyan of the generated image I_g_ and the feature vector *m*_*P*_ of the *i*th king image in the similar image probationer decoy *P*, the similarity between the generated image *I*_g_ and the *i*th real image in the similar image candidate Bethesda *P* is *S*_*i*_ = ‖ *mI*_g_ · *mP*_*i*_ ‖ ‖ ‖Mikoyan ‖*t*‖‖*mP*_*i*_ ‖, we calculate the cosine similarity between the variety similarity in the similar actor pool *P* and all realism programs. Afterward, we arrange the similarity motivation in descending order to keep the top *N* royal images. The personality *SI*_g_ of the generated appearance *I*_g_ is arguably the disgrace of the top *N* concept similarity scores: *SI*_g_ = 1 *N*∑_*i*_^*N*^*s*_*i*_ + *S*_t_.

## 4. Experimental Results and Analysis

This section evaluates the proposed reconstruction image configuration evaluation algorithm by leveraging a public GAN dataset and a generated portrait feature evaluation dataset. The experimental platform is Intel(R) Xeon(R) Gold5218CPU @2.30 GHz information processing system. Tesla P100 GPU is used for fork drag and drop, wherein the language of the prospectus is Python3.6. We believe that the framework is Pytorch1.5, and the unified estimation is built upon the CUDA10.1. All similar features are extracted by the Universal Design Education of ImageNet. The NN-GIQA process in this disembodied federated Flickr-Faces-HQ (FFHQ) dataset and the NN *N* in the Cityscapes dataset are fixed to 1, while the farthest neighbor *N* in the LSUN-cat is set to 3500.

The experiments leverage the GAN classic datasets FFHQ, LSUN, Cityscapes, and the generative image quality assessment dataset LGIQA to evaluate the conversation-generated portrait quality assessment method. FFHQ is a grumpy air dataset that embrace 70,000 plentifully specify existence similarities in PNG reformatting with 1024 × 1024 persistence. Imagery is plentiful and diverse with deference to age, ethnicity, and figures. Meanwhile, there are many variations in facial attribution. It features distinct age, gender, race, skin markers, expressions, face shape, hairstyle, and facial pose. Characters from this data are set with common glasses, sunglasses, gibus, beard accessories, scars, and other peripheral accessories. LSUN is a giant disk appearance dataset compiled for deep learning. It mainly includes 10 exhibition categories, such as cubiculum, kitchen, live latitude, and classroom, and 20 visual categories, such as miauler, dicky, airplane, and electric bus. Each scenic category contains about one million tags. Also, each opposition category contains over one million tickets. Cityscapes is a new rich ascent dataset containing scene images from 50 different cities. It contains 5000 manually annotated images whose resolution is 1024 × 2048. It also contains 20,000 coarse glaze castings. These are accurately annotated images containing 2975 educational representations, 500 verification appearances, and 1525 test displays. LGIQA is a dataset collected by Gu et al. It is annotated by multiple clod observers, the three data subsets embodied are LGIQA-FFHQ, LGIQA-LSUN-cat, and LGIQA-Cityscapes. The three datasets are initially comprised of 1500 image pairs from PGGAN-propagate semblance, StyleGAN-cause cast, and Kerçek show. Class observers exhibit image damage, preventing them from adopting better quality images in the program pair, discarding concepts they disagreed with among the three data set. It can beautify LGIQA-FFHQ data with 974 images in flight and LGIQA-FFHQ data with 1206 images suit. LSUN-mouser dataset and LGIQA-Cityscapes dataset contain 1102 image in total.

In order to more intuitively evaluate the estimation implementation of the algorithm, we show the images in the LGIQA dataset and their NN-GIQA reasons. The top 5 images of replicas are displayed with the highest ranking counts in each subset of LGIQA obtained using NN-GIQA. Asher top 5 shows the images with the lowest ranking reasons for pictures in each of LGIQA. The data idol spans in the annotations and their NN-GIQA fees. The image pairs are from port to vertical images from LGIQA-FFHQ, LGIQA-LSUN-cat, and LGIQA-Cityscapes, respectively. Each double of similarities is the kind corresponding to the observer's annotation. Higher conception disposition displays are verified on the sinister, whereas semblance with lower image prosecute charged are confirm upright. The bottom half of the portrait is its NN-GIQA score. Comparing the high-level actors in Table 1 with the blaze-sort replicas, and the likeness pairs and their corresponding NN-GIQA scores in Table 2, it is manifest that the method in this no-being competent the humane vision. In practice, the plant ranking results are uniform with human evaluations.

In order to verify the accuracy and operational efficiency of the rules in this experiment, we have concluded from experiencing the native copywriting temperament evaluation method and the subsequent conversation reason casting temperament evaluation method. The evaluation method is proposed by Gu et al. It is pervasively utilized to score the GIQA algorithm program proposed in this article. We conduct the correctness evaluation of the algorithm rules, obtain the real motivation of the generated portraits through NN-GIQA, pair the quality of each group of images, and check whether the overall results are consistent with the labels raised by the human evaluation. We can thus obtain the accuracy of the algorithm program, and further criticize pictures by the accuracy of the algorithm. Whether the industry evaluation method is in line with human visual perception is a key factor. We naturally reveal the natural evaluation laws: deciding to refine the no-reference image quality evaluation methods, such as DeepIQA [3], RankIQA [13], and NIMA [14]. The DeepIQA model and the NIMA model are discriminated on the dataset. We use the degradation strategy of RankIQA and Direct fine-tuning. Then we leverage the IQA algorithm to train and experiment on the dataset. Generated image quality assessment methods are used. Both the scholarship-supported and data-based methods are experimented. Methods to learn support end regression IR-GIQA for generating projected character scores are leveraged by the convolutional neural network model. We use a binary classifier to shape whether the generated image is BCGIQA. Meanwhile, a second-hand manifold binary classifier is trained to learn for propagating image quality ratings. Data-backed methods are called the SGM-GIQA, which applies the Gaussian examples to obtain probability assignments for the royal data, and subsequently we rate the quality of reproduced images.

We further apply the proposed GMM-GIQA, which uses Gaussian mixtures to evaluate probability distributions over real data to evaluate the quality of the generated images. We further experimentally compare GMM-GIQA, which uses a Gaussian mixture fork to capture the probability distribution of the real data and evaluate the quality of the growth picture. We also compare with KNN-GIQA, which produces the contrast between an idol and its KNN. We evaluate the conceptual temperament of a variety. Table 1 summarizes the similarity termination for the accuracy of different replicated character-evaluation methods on the LGIQA dataset. Through comparison, it can be observed that the evaluation accuracy of the NN-GIQA method is higher than that of the natural portrait attribute evaluation method on the LGIQA dataset. This indicates that the evaluation technique of natural appearance ranking is inconsistent with the evaluation method of visual quality prediction. According to the LGIQA-Cityscapes dataset, the accuracy of NN-GIQA is higher than most learning-enabled methods and close to data-based methods. Experimental results verified the accuracy of the method for the quality of conception copies. Besides, the evaluation process is consistent with human visual perception. In addition, the authenticity of our method is over 80% on different data adjustments. This can show the generalization ability of the method.

To average metric calculated to measure the progress of Similar Name Preservation (CND) features based on the harbinger effect of color display quality assessment models. We also conduct the ablative study on a series of features, including the CND, gradient, and luminance on the TID2008 dataset. Here, the CNCI standard utilizes only the CND form, walking form, and gloss features. Simultaneously, the Special Report on the Ocean and Cryosphere in a Changing Climate (SROCC) importance that can be performed when the three features are combined in a set and all three features are used collaboratively. It can be observed that the maximum SROCC value can be calculated by using the simultaneous tense of the above features. Since HVS focuses on gloss human visual perception rather than excuse perception, the slop formed by second-hand light-only grooves and second-hand brightness-only shapes perform slightly better than second-hand CND-only features. However, it can be observed in Table 2 that after the adoption of the CND after feature engineering, the evaluation performance of the GAN-generated image has been remarkably improved. This can demonstrate that the color feature is the most informative in the perceptual category competition among the aforementioned color descriptors.

## 5. Conclusions

In this article we proposed a GAN-generated image quality evaluation method based on the NN algorithm. We realize the quality evaluation of images generated by different GAN models on different datasets. The experimental results have shown that the method in this article performs well on multiple datasets. Also, the obtained evaluation and the results are consistent with the human evaluation results. Compared with the existing quality models, the method in this article greatly improves the computational efficiency and the computational accuracy.

However, when the generated image boundary is partially distorted, the generated image quality evaluation results calculated by our method is still not perfect than those based on humans. There will be differences with the human evaluation results, and this issue will be our future work.

## Figures and Tables

**Table 1:** Different IQA algorithms on LGIQA data sets.

Data set	LGIQA-FFHQ	LGIQA-LSUN-cat	LGIQA-Cityscapes
DeepIQA	0.674	0.674	0.584
RankIQA	0.732	0.694	0.674
MIMA	0.674	0.684	0.721
IR-GIQA	0.743	0.712	0.683
BC-GIQA	0.683	0.772	0.732
MBC-GIQA	0.682	0.658	0.732
SGM-IQA	0.645	0.683	0.684
GMM-GIQA	0.703	0.583	0.704
KNN-GIQA	0.741	0.793	0.784
Ours	0.793	0.902	0.822

**Table 2:** Running time cost of different IQA methods.

Data set	LGIQA-FFHQ (s)	LGIQA-LSUN-cat (s)	LGIQA-Cityscapes (s)
GMM-GIQA	1343.212	1832.332	1843.221
KNN-GIQA	344.321	1032.106	894.342
NN-GIQA	99.832	432.121	564.443

## Data Availability

Data supporting this research article are available from the corresponding author or first author on reasonable request.
